The article "A Low-Cost Multistage Cascaded Adaptive Filter Configuration for Noise Reduction in Phonocardiogram Signal" was published in 2022. Journal: J Healthc Eng.

# A Low-Cost Multistage Cascaded Adaptive Filter Configuration for Noise Reduction in Phonocardiogram Signal

**DOI:** 10.1155/2022/3039624

**Published:** 2022-04-30

**Authors:** S. Hannah Pauline, Samiappan Dhanalakshmi, R. Kumar, R. Narayanamoorthi, Khin Wee Lai

**Affiliations:** ^1^Department of Electronics and Communication Engineering, College of Engineering and Technology, Faculty of Engineering and Technology, SRM Institute of Science and Technology, SRM Nagar, Kattankulathur 603203, Kanchipuram, Chennai, Tamil Nadu, India; ^2^Department of Electrical and Electronics Engineering, College of Engineering and Technology, Faculty of Engineering and Technology, SRM Institute of Science and Technology, SRM Nagar, Kattankulathur 603203, Kanchipuram, Chennai, Tamil Nadu, India; ^3^Department of Biomedical Engineering, Faculty of Engineering, Universit Malaya, Kuala Lumpur 50603, Malaysia

## Abstract

Phonocardiogram (PCG), the graphic recording of heart signals, is analyzed to determine the cardiac mechanical function. In the recording of PCG signals, the major problem encountered is the corruption by surrounding noise signals. The noise-corrupted signal cannot be analyzed and used for advanced processing. Therefore, there is a need to denoise these signals before being employed for further processing. Adaptive Noise Cancellers are best suited for signal denoising applications and can efficiently recover the corrupted PCG signal. This paper introduces an optimal adaptive filter structure using a Sign Error LMS algorithm to estimate a noise-free signal with high accuracy. In the proposed filter structure, a noisy signal is passed through a multistage cascaded adaptive filter structure. The number of stages to be cascaded and the step size for each stage are adjusted automatically. The proposed Variable Stage Cascaded Sign Error LMS (SELMS) adaptive filter model is tested for denoising the fetal PCG signal taken from the SUFHS database and corrupted by Gaussian and colored pink noise signals of different input SNR levels. The proposed filter model is also tested for pathological PCG signals in the presence of Gaussian noise. The simulation results prove that the proposed filter model performs remarkably well and provides 8–10 dB higher SNR values in a Gaussian noise environment and 2-3 dB higher SNR values in the presence of colored noise than the existing cascaded LMS filter models. The MSE values are improved by 75–80% in the case of Gaussian noise. Further, the correlation between the clean signal and its estimate after denoising is more than 0.99. The PSNR values are improved by 7 dB in a Gaussian noise environment and 1-2 dB in the presence of pink noise. The advantage of using the SELMS adaptive filter in the proposed filter model is that it offers a cost-effective hardware implementation of Adaptive Noise Canceller with high accuracy.

## 1. Introduction

The phonocardiogram signal [1] contains important information about the heart's operations and is used to detect various heart disorders [2]. However, recording PCG signals and other biomedical signals [3, 4] is very challenging since they are susceptible to environmental noise apart from the other noise signals [5]. As a result, denoising of PCG signals is a mandatory requirement before its analysis [6]. Nevertheless, denoising a PCG signal to increase signal quality by removing the background noise is difficult. The accuracy of results is determined by the performance of denoising algorithms used, which diminishes as the noise level rises [7]. Various PCG signal denoising approaches have been proposed in the literature based on the time and frequency domain [8]. Frequency domain methods are preferred since they contain adequate information on the spectral characteristics of the PCG signal components [9]. Among the frequency domain approaches, the most commonly used techniques are Empirical Mode Decomposition (EMD) [10, 11], Variational Mode Decomposition (VMD) [12], Singular Spectrum Analysis (SSA) [13], and Tunable Q-Wavelet Transform [14]. Although these techniques give an efficient performance, the computational time is high. Compared to all the proposed techniques for PCG signal denoising, the Discrete Wavelet Transform (DWT) [15, 16] is more effective and performs better in a noisy environment. However, it requires a predefined basis function to produce optimal SNR values. In this paper, we have explored the possibility of applying the Adaptive Noise Cancellation technique using adaptive filters, which is predominantly used for signal denoising in telecommunication to PCG signal denoising. Adaptive filters provide the best estimate of clean signals with automatic performance adaptation. Adaptive algorithms employed in adaptive filters track the dynamic variations in the signal and modify their behavior according to the input signal; therefore, they are used in several applications, including echo [17, 18] and noise cancellation [19], noise reduction [20], signal enhancement [21, 22] adaptive equalization [23], and line enhancement [24]. The fundamental Adaptive Noise Canceller is depicted in Figure 1.

The primary input signal provided to the ANC is the noisy signal *d*(*n*) defined as

(1) $$\begin{array}{c} d\left(n\right)=s\left(n\right)+v\left(n\right), \end{array}$$

where *s*(*n*) is the noise-free signal and *v*(*n*) is the added noise signal. *s*(*n*) and *v*(*n*) are not time correlated to each other, and the input signal to the filter *x*(*n*) is a noise signal in time correlated to *v*(*n*). The adaptive filter gives the replica of the noise signal and $\hat{v}\left(n\right)$ as

(2) $$\begin{array}{c} y\left(n\right)=w^{T}\left(n\right)x\left(n\right), \end{array}$$

where **w**(*n*)=[*w*_0_, *w*_1_,…*w*_*M*−1_]^*T*^ and **x**(*n*)=[*x*_0_(*n*), *x*_1_(*n* − 1),…*x*_*M*−1_(*n* − *M*+1)]^*T*^ are weights of the filter and its input, respectively, *M* is the order of filter, and the error signal is computed as

(3) $$\begin{array}{c} e\left(n\right)=d\left(n\right)-y\left(n\right)\\ =d\left(n\right)-\hat{v}\left(n\right), \end{array}$$

such that the effect of noise is minimal. The efficiency of the adaptive filter is improved by using suitable algorithms like LMS and its variants. Due to its feasible implementation and robustness, the LMS adaptive algorithm [25] is commonly used. Sign Error LMS adaptive algorithm has less number of computations than the LMS algorithm but to achieve a good performance, smaller step size should be used. The SE LMS algorithm, however, suffers from low convergence speeds. The convergence speed can be improved and the steady-state MSE minimized by optimizing the adaptive filter structure [26] as suggested by several researchers. The cascaded adaptive filter structure was first proposed by Ahmed et al. [27] for the detection of multiple sinusoids. The cascaded filter structure is effectively employed to enhance and track multiple sinusoids. A cascaded structure of the FIR filter proposed by Prandoni and Vetterli [28] for adaptive linear prediction proves that, compared to a single-stage filter, a cascaded structure converges faster to an optimal predictor. The major advantage pointed out in [28] is the computational efficiency of the cascaded adaptive filter structure. For lossless compression of audio signals, several techniques have been proposed in literature based on Laplacian distribution [29], decoupled approach [30], context model [31], linear transforms [32], and linear prediction [33]. However, the nonstationary feature of audio signals requires the use of an adaptive filtering approach [34] for lossless audio coding since adaptive filters provide good tracking capability. A cascade combination of higher-order LMS filter and lower-order RLS filter proposed by Yu and Ko [35] is used as a predictor for lossless audio coding. This cascaded RLS-LMS predictor provides faster convergence and superior prediction gain as it uses a cascade combination of low complexity LMS filter and high converging RLS filter models. For MPEG-4 lossless audio coding [36], the cascaded RLS-LMS predictor attains the best compression ratio. In ANC (Active Noise Cancellation) systems, the Filtered × Least Mean Square (FxLMS) algorithm [37] is widely applied for efficient noise cancellation. Nevertheless, the FxLMS algorithm's steady-state performance is affected by the presence of uncorrelated noise at the error sensor. The cascaded adaptive filtering approach proposed by [38] is successful in preventing ANC filter coefficient oscillation, thus improving the convergence speed. In mechanical and automobile engineering, denoising engine vibrations and other types of noise are of interest to several researchers. Median filtering [39] and wavelet packet threshold denoising [40] are prominent among the existing noise and vibration denoising techniques. More recently, a combination of median filtering and wavelet packet denoising has been effectively used for vibration signal denoising [41]. Adaptive filtering is applied to active noise and control due to its self-tuning capability. For engine noise suppression [42], the use of cascaded LMS adaptive filter models shows that the adaptation of the filter speed is improved. Recently Multistage Adaptive LMS (MSA-LMS) algorithm proposed by [43] has been applied to active vibration and noise control systems and given remarkable performance for signals with complex frequency spectra. Multilevel Adaptive Noise Cancellers have proven to be very effective in AE- (Acoustic Emission-) based methods to detect rail defects. The simple wavelet hard threshold denoising method [44] causes a loss of useful information and cannot change according to the noise signal variations. To eliminate complex noise and retain the information signal at fast speeds, multilevel noise cancellation based on SANC (Self-Adaptive Noise Cancellation) and ANC is proposed by Zhang et al. in [45], which proves to provide good noise suppression capabilities. Adaptive filtering plays a significant role in biomedical engineering to remove noise and artifacts from ECG signals. The presence of artifacts is one of the crucial challenges in ambulatory ECG monitory systems. For motion artifact removal, several techniques are proposed, and they can be categorized into two, namely, adaptive filtering and Blind Source Separation (BSS) [46]. Although the BSS approach can provide good filtering performance, the adaptive filtering-based approach has a more practical advantage due to its computational simplicity and adaptability to meet the hardware requirements of the system [47]. The efficient removal of artifacts from ambulatory ECG signals [47] is achieved using a cascaded LMS adaptive filter model. Efficient elimination of multiple noise signals from ECG signal [48] is obtained with high output SNR value and faster convergence speed by using a multistage modified NLMS algorithm. A novel 2-stage cascaded LMS adaptive filter configuration is proposed by Dixit in [49] and a 3-stage [50] cascaded LMS adaptive filter by Maurya for Adaptive Noise Cancellation. The proposed cascaded adaptive filter architectures are tested for denoising sinusoidal signals. It has been proved that, compared to traditional LMS adaptive filters, the 2-stage and 3-stage cascaded LMS adaptive filter architectures proposed for Adaptive Noise Cancellation provide better efficiency in terms of SNR and MSE performance.

The above studies show that, for several applications, including Active Noise Control, signal enhancement, linear prediction, noise cancellation, and suppression, the cascaded adaptive filter model performs better than the conventional single-stage adaptive filter in convergence speed and MSE. The above studies have not explored the possibility of varying the number of cascaded filter stages required for the ANC to reach its optimal performance in terms of MSE and convergence speed. The number of cascaded stages and the step size for each stage are fixed in the above-proposed structures. In this work, we propose a novel Variable Stage Cascaded Sign Error (SE) LMS adaptive filter structure wherein the number of filter stages to be cascaded to give optimal performance in steady-state MSE is selected automatically. In contrast, in the existing cascaded filter models, the number of cascaded stages is fixed. To obtain a faster convergence speed, the step size should be adjusted at each stage. The number of cascaded filter stages and the step size for each stage are adjusted automatically to achieve optimal performance regarding steady-state MSE and convergence speed in the proposed filter structure. We have also analyzed the behavior of the proposed filter model using a fixed step size for all the stages. The novelty of the proposed Variable Stage Cascaded SE LMS adaptive filter model is summarized as follows:

- Using Sign Error LMS adaptive filter in a cascaded configuration to denoise PCG signals to reduce the hardware cost.
- Automatic adjustment of an optimal number of stages to obtain efficient performance in terms of convergence speed of steady-state MSE.
- Automatic adjustment of the step size of the adaptive filter at each stage ANC to improve the convergence speed.

Compared to the existing signal denoising techniques, the primary advantage of the proposed filter model is the reduction in computational complexity. The proposed filter model employs the SE LMS [51] algorithm for adaptation, which requires a minimum number of computations and provides a low-cost and straightforward implementation of a hardware processor for efficient denoising of PCG signals. Further, the automatic addition of an optimal number of stages provides a minimum MSE value, and the adjustment of step size at each stage helps achieve faster convergence speeds. The results indicate that the proposed Variable Stage (VS) Cascaded Sign Error LMS adaptive filter model provides minimum steady-state MSE and faster convergence speed. The proposed Variable Stage Cascaded SE LMS adaptive filter model is detailed in Section 2.  Section 3 includes the MATLAB simulation results, thus verifying the proposed method's effectiveness, the results are discussed in Section 4, and a conclusion with the future scope is included in Section 5.

## 2. Proposed Variable Stage (VS) Cascaded Sign Error LMS Adaptive Filter Structure

The use of the LMS adaptive algorithm in conventional ANC systems leads to a computationally simpler structure with superior robustness and stability. LMS algorithm is more suited for software implementation. The Sign Error LMS algorithm, a variant of the LMS algorithm, gives a computationally more straightforward and cost-effective implementation of Adaptive Noise Cancellation. It suffers from slow convergence and large steady-state MSE compared to the LMS algorithm. The performance degradation can be avoided by using a smaller step size than the LMS algorithm. Also, the cascaded adaptive filter structure employed in the ANC system helps to reduce the steady-state MSE and increase its convergence speed. We proposed a multistage cascaded configuration of adaptive filters using the Sign Error LMS adaptation algorithm at each stage. The features of the proposed Variable Stage (VS) Cascaded Sign Error (SE) LMS adaptive filter model are as follows:

- The number of stages to be cascaded to provide optimal steady-state MSE and convergence speed is automatically varied.
- The step size of the Sign Error LMS adaptation algorithm is adjusted at each stage automatically to improve the convergence speed of the steady-state MSE.

Figure 2 depicts the block diagram representation of the proposed Variable Stage (VS) Cascaded Sign Error (SE) LMS adaptive filter model, and the schematic diagram is depicted in Figure 3. As depicted in Figure 3, the primary input signal to stage I ANC is the noisy signal *d*_1_(*n*)=*s*(*n*)+*v*(*n*), and the reference input signal is the noise signal *v*′(*n*) correlated to *v*(*n*). The primary input signal to stage II ANC *d*_2_(*n*) is the output error signal *e*_1_(*n*) of stage I, and the reference input signal to stage II adaptive filter *x*_2_(*n*) is the residual reference noise signal from stage I, *x*_1_(*n*) − *y*_1_(*n*). In the same way, the error signal of each stage ANC *e*_*i*_(*n*) is given to the next stage ANC as its primary input signal *d*_*i*+1_(*n*), and the reference noise input to the *i*^*th*^ stage *x*_*i*_(*n*) is the residual reference noise *x*_*i*−1_(*n*) − *y*_*i*−1_(*n*) from the preceding (*i* − 1)^th^ stage ANC. The number of stages to be cascaded to attain optimal performance is adjusted automatically, and the step size of the adaptive filter at each stage is controlled automatically.

The parameters of stage I ANC using the Sign Error LMS algorithm are as follows:

Primary input signal

(4) $$\begin{array}{c} d_{1}\left(n\right)=s\left(n\right)+v\left(n\right). \end{array}$$

Reference input signal

(5) $$\begin{array}{c} x_{1}\left(n\right)=v^{\prime }\left(n\right). \end{array}$$

Filter output

(6) $$\begin{array}{c} y_{1}\left(n\right)=w_{1}^{T}\left(n\right)x_{1}\left(n\right)\\ =w_{1}^{T}\left(n\right)v^{\prime }\left(n\right)\\ =\hat{v}\left(n\right), \end{array}$$

where **w**_1_(*n*)=[*w*_0_, *w*_2_,…*w*_*M*−1_]^*T*^ and **x**_1_(*n*)=[*x*_0_(*n*), *x*_1_(*n* − 1),…*x*_*M*−1_(*n* − *M*+1)]^*T*^ are weights of the filter and its input, respectively, at stage I, and *M* is the filter order.

Weight update equation

(7) $$\begin{array}{c} w_{1}\left(n+1\right)=w_{1}\left(n\right)+\mu_{1\text{SELMS}}\mathrm{sgn}\left[e_{1}\left(n\right)\right]v^{\prime }\left(n\right), \end{array}$$

where *μ*_1SELMS_ is the step size of Sign Error LMS filter.

Output error

(8) $$\begin{array}{c} e_{1}\left(n\right)=d_{1}\left(n\right)-y_{1}\left(n\right)\\ =s\left(n\right)+v\left(n\right)-\hat{v}\left(n\right)\\ =s\left(n\right)+\Delta v\left(n\right), \end{array}$$

where $\Delta v\left(n\right)=v\left(n\right)-\hat{v}\left(n\right)$ is the noise signal to be minimized.

The parameters of stage II ANC are as follows:

Primary input signal

(9) $$\begin{array}{c} d_{2}\left(n\right)=e_{1}\left(n\right)\\ =d_{1}\left(n\right)-\hat{v}\left(n\right)\\ =s\left(n\right)+\Delta v\left(n\right). \end{array}$$

Reference input signal

(10) $$\begin{array}{c} x_{2}\left(n\right)=x_{1}\left(n\right)-y_{1}\left(n\right)=v^{\prime }\left(n\right)-\hat{v}\left(n\right)=\Delta v^{\prime }\left(n\right). \end{array}$$

Filter output

(11) $$\begin{array}{c} y_{2}\left(n\right)=w_{2}^{T}\left(n\right)x_{2}\left(n\right)\\ =w_{2}^{T}\left(n\right)\Delta v^{\prime }\left(n\right)\\ =\Delta \hat{v}\left(n\right). \end{array}$$

Weight update equation

(12) $$\begin{array}{c} w_{2}\left(n+1\right)=w_{2}\left(n\right)+\mu_{2\text{SELMS}}\mathrm{sgn}\left[e_{2}\left(n\right)\right]\Delta v^{\prime }\left(n\right). \end{array}$$

Output error

(13) $$\begin{array}{c} e_{2}\left(n\right)=d_{2}\left(n\right)-y_{2}\left(n\right)=s\left(n\right)+\Delta v\left(n\right)-\Delta \hat{v}\left(n\right)=s\left(n\right)+\delta v\left(n\right), \end{array}$$

where $\delta v\left(n\right)=\Delta v\left(n\right)-\Delta \hat{v}\left(n\right)$ is the remaining noise to be minimized. The number of stages to be cascaded is adjusted till the *L*^th^ optimal stage is reached. The parameters of stage L ANC are as follows:

Primary input signal

(14) $$\begin{array}{c} d_{L}\left(n\right)=e_{L-1}\left(n\right)\\ =s\left(n\right)+\rho v\left(n\right), \end{array}$$

where *ρv*(*n*) is a minimal noise.

Reference input signal

(15) $$\begin{array}{c} \begin{array}{c} x_{L}\left(n\right)=x_{L-1}\left(n\right)-y_{L-1}\left(n\right)\\ =\rho v^{\prime }\left(n\right). \end{array} \end{array}$$

Filter output

(16) $$\begin{array}{c} y_{L}\left(n\right)=w_{L}^{T}\left(n\right)x_{L}\left(n\right)\\ =w_{L}^{T}\left(n\right)\rho v^{\prime }\left(n\right)\\ =\rho \hat{v}\left(n\right). \end{array}$$

Weight update equation

(17) $$\begin{array}{c} w_{L}\left(n+1\right)=w_{L}\left(n\right)+\mu_{\text{LSELMS}}\mathrm{sgn}\left[e_{L}\left(n\right)\right]x_{L}\left(n\right). \end{array}$$

Output error

(18) $$\begin{array}{c} e_{L}\left(n\right)=d_{L}\left(n\right)-y_{L}\left(n\right)\\ =s\left(n\right)+\rho v\left(n\right)-\rho \hat{v}\left(n\right)\approx s\left(n\right), \end{array}$$

where $\rho v\left(n\right)-\rho \hat{v}\left(n\right)=\eta v\left(n\right)$, where *η* is a very small quantity. The above analysis ensures that, by adjusting the number of filter stages to its optimum value *L*=*L*_*opt*_, the noise is minimized further, and thus steady-state MSE reduces significantly. The employment of automatic stage selection gives optimal performance in steady-state MSE, and the convergence speed is further improved by using different step size for each stage. The appropriate step size at each stage is also selected automatically. The closest estimate of the noise-free signal is obtained as the filter reaches its optimal stage. This signal *e*_*L*_(*n*) ≈ *s*(*n*) is closely related or in time correlated to the clean signal *s*(*n*).

### 2.1. Mean Square Error (MSE)

The error signal at the optimal stage is

(19) $$\begin{array}{c} e_{L}\left(n\right)=d_{L}\left(n\right)-y_{L}\left(n\right)\\ =s\left(n\right)+v\left(n\right)-y_{1}\left(n\right)-y_{2}\left(n\right)-\ldots -y_{L}\left(n\right)\\ =s\left(n\right)+v\left(n\right)-\left[y_{1}\left(n\right)+y_{2}\left(n\right)+\cdots +y_{L}\left(n\right)\right]. \end{array}$$

At the optimal stage *L* of the ANC, $y_{1}\left(n\right)+y_{2}\left(n\right)+\cdots +y_{L}\left(n\right)=\tilde{v}\left(n\right)$ (replica of *v*(*n*)) and the MSE is denoted as

(20) $$\begin{array}{c} E\left[{\left|e_{L}\left(n\right)\right|}^{2}\right]=E\left[{\left|s\left(n\right)\right|}^{2}\right]+E\left[{\left|v\left(n\right)-\tilde{v}\left(n\right)\right|}^{2}\right]\\ -2E\left[\left|s\left(n\right)\left(v\left(n\right)-\tilde{v}\left(n\right)\right)\right|\right]\\ =E\left[{\left|s\left(n\right)\right|}^{2}\right]+E\left[{\left|v\left(n\right)-\tilde{v}\left(n\right)\right|}^{2}\right]\\ -2E\left[\left|s\left(n\right)v\left(n\right)\right|\right]+2E\left[\left|s\left(n\right)\tilde{v}\left(n\right)\right|\right]. \end{array}$$

The following equation is obtained due to the uncorrelation between noise *v*(*n*) and the information signal *s*(*n*).

(21) $$\begin{array}{c} 2E\left[\left|s\left(n\right)v\left(n\right)\right|\right]=0. \end{array}$$

Meanwhile, *s*(*n*) and output of the adaptive filter $\hat{v}\left(n\right)$ are also uncorrelated; hence, the following is stated:

(22) $$\begin{array}{c} 2E\left[\left|s\left(n\right)\tilde{v}\left(n\right)\right|\right]=0. \end{array}$$

Inserting equations (21) and (22) in (20),

(23) $$\begin{array}{c} E\left[{\left|e_{L}\left(n\right)\right|}^{2}\right]=E\left[{\left|s\left(n\right)\right|}^{2}\right]+E\left[{\left|v\left(n\right)-\tilde{v}\left(n\right)\right|}^{2}\right]. \end{array}$$

Further, it is observed that the best replica of the information signal *s*(*n*) is achieved as the term $E\left[{\left|v\left(n\right)-\tilde{v}\left(n\right)\right|}^{2}\right]$ is minimized. It means that, at the optimal filter stage *L*, *y*_1_(*n*)+*y*_2_(*n*)+⋯+*y*_*L*_(*n*) is as close to *v*(*n*) as possible, and hence, $E\left[{\left|v\left(n\right)-\tilde{v}\left(n\right)\right|}^{2}\right]$ is minimized. The equation is represented as

(24) $$\begin{array}{c} \left[y_{1}\left(n\right)+y_{2}\left(n\right)+\cdots +y_{L}\left(n\right)\right]\approx v\left(n\right). \end{array}$$

The above analysis proves that the noise signal can be removed from the input signal *d*_1_(*n*) by adjusting the number of stages of the filter, and *O*(*n*) represents the denoised signal from the ANC.

(25) $$\begin{array}{c} O\left(n\right)=e_{L}\left(n\right)\approx s\left(n\right). \end{array}$$

From the above analysis, we infer that the denoised signal *O*(*n*) is obtained as the number of stages in the cascaded filter structure approaches its optimal value.

### 2.2. Automatic Stage Selection Control Logic

The above analysis concludes that the MSE value reaches its minimum only at the filter's optimal stage. To calculate the optimum filter stage, we estimate the Pearson cross-correlation function between the error signal of each stage *e*_*i*_(*n*) and the reference input noise signal *v*′(*n*). We have assumed that the reference noise signal *v*′(*n*) to stage I adaptive filter is correlated to the additive noise signal *v*(*n*) but is uncorrelated to the clean signal *s*(*n*). The error output of each stage ANC is an estimate of the clean signal; that is, $e_{i}\left(n\right)=\hat{s}\left(n\right)$; therefore, the correlation between *e*_*i*_(*n*) and *v*′(*n*) reduces as the filter reaches its optimal stage. The estimated correlation function between *e*_*i*_(*n*) and *v*′(*n*) is defined as

(26) $$\begin{array}{c} \rho_{e_{i},v^{\prime }}=\frac{\text{Cov}\left(e_{i},v^{\prime }\right)}{\sigma_{e_{i}}\sigma_{v^{\prime }}}, \end{array}$$

where *ρ*_*e*_*i*_,*v*′_ is the Pearson product-moment correlation coefficient, Cov(*e*_*i*_, *v*′) is the covariance of variables *e*_*i*_ and *v*′, and *σ*_*e*_*i*__ and *σ*_*v*′_ are the standard deviation of *e*_*i*_ and standard deviation of *v*′. In the proposed method, *e*_*i*_(*n*) is the estimate of the clean signal at each stage and *v*′(*n*) is the reference noise signal used at stage I. Since we have presumed that the information signal *s*(*n*) and the added noise are uncorrelated, the value of *ρ*_*e*_*i*_,*v*′_ should be low. The estimated correlation function *ρ*_*e*_*i*_,*v*′_ is investigated at each stage, and further adaptive filter stages are added until the value of *ρ*_*e*_*i*_,*v*′_ reaches a minimal threshold value at the optimal cascaded filter stage.

### 2.3. Variable Step Size for Each Stage

The performance of the Sign Error LMS algorithm can be as good as LMS algorithms if we select a step-size value lower than the LMS algorithm. Thus, the step size of the Sign Error LMS algorithm is selected based on the LMS algorithm. The major challenge with the LMS algorithm is the choice of step size. A significant step size results in fast adaptation but provides a large excess Mean Square Error (excess MSE). A too-large step size will lead to a loss of stability. On the other hand, a too-small step-size result in slow convergence even though the excess MSE is minimum. The upper bound for step size in order to sustain the stability of the LMS algorithm is given by [52]

(27) $$\begin{array}{c} 0<\mu <\frac{2}{\lambda_{\max}}, \end{array}$$

where *μ* is the step size and *λ*_max_ is the largest eigenvalue of the autocorrelation matrix of the input signal *x*(*n*). In the proposed filter model, the input to each filter stage is the residual reference noise from the previous stage; hence, different input signal is given to the filter at each stage. Therefore, instead of using the same step-size value for all the stages, using different step size at each stage improves the filter's speed of adaptation. We select a fixed value of step size for stage I adaptive filter by first finding *μ*_1max_ and then selecting the step size for the LMS algorithm using equation (27) as *μ*_1*LMS*_ ≤ *μ*_1max_. Then, we divide this value by *x*=10 to obtain the step size of Sign Error LMS at stage I.

(28) $$\begin{array}{c} \mu_{1\text{SELMS}}=\frac{\mu_{1\text{LMS}}}{x}\\ =\frac{\mu_{1\text{LMS}}}{10}, \end{array}$$

where *x*=10 is selected by using the trial and error method. At stage II, the input to the adaptive filter is *x*_2_(*n*)=*x*_1_(*n*) − *y*_1_(*n*), which means that the input signal to the filter changes at each stage and based on the input, the upper bound for step size also changes. At stage II, we calculate the upper bound of step size *μ*_2max_ for the LMS algorithm using equation (27). Then, the value of *μ*_2max_ is compared with *μ*_1max_. If *μ*_2max_ > *μ*_1max_, then a higher step size is desired for the stage II adaptive filter. Therefore, we set *μ*_2*LMS*_=*μ*_1*LMS*_*∗k* and

(29) $$\begin{array}{c} \mu_{2\text{SELMS}}=\frac{\mu_{1\text{LMS}}}{10}*k\\ =\mu_{1\text{SELMS}}*k, \end{array}$$

where *k* is a constant selected by trial and error method. Otherwise, if *μ*_2max_ < *μ*_1max_, then a smaller step size is required, so we adjust *μ*_2*LMS*_=*μ*_1*LMS*_*∗*1/*k* and

(30) $$\begin{array}{c} \mu_{2\text{SELMS}}=\frac{\mu_{1\text{LMS}}}{10}*\frac{1}{k}\\ =\mu_{1\text{SELMS}}*\frac{1}{k}. \end{array}$$

In this way, the step size for the filter at each stage is adjusted as

(31) $$\begin{array}{c} \mu_{i}=\left\{\begin{array}{cc} \mu_{i-1}*\left(k\right), & \mu_{{\text{max}}_{i}}>\mu_{{\text{max}}_{i-1}},\\ \mu_{i-1}*\left(\frac{1}{k}\right), & \mu_{\max_{i}}<\mu_{{\text{max}}_{i-1}}, \end{array}\right. \end{array}$$

where *μ* denotes the step size of SE LMS filter at *i*^th^ and (*i* − 1)^th^ stage, *μ*_max_ denotes the upper bound of step size for LMS filter, and ′*k*′ is a constant value that varies between 1 and 2; selecting the ′*k*′ value is crucial for the convergence of the filter stage. The proposed Variable Stage Cascaded SE LMS adaptive filter model that uses variable step size for each stage has a faster convergence speed than fixed step size for all stages.

By automatically adjusting the number of cascaded stages and the step size at each stage, the steady-state MSE reduces, and convergence speed is improved. Proposed Variable Stage Cascaded SE LMS adaptive filter model used for Adaptive Noise Canceller is summarized in Algorithm 1.

## 3. Results

The performance of the proposed Variable Stage Cascaded SE LMS adaptive filter is tested for fetal PCG (PhonoCardioGram) signal taken from the Shiraz University Fetal Heart Sounds Database (SUFHSDB) [53, 54]. A fetal PCG signal (f1) of duration 2 s was taken from the SUFH database, sampled at 16 kHz. The signal is corrupted by Gaussian and colored (pink) noise of input SNR +4 and −4. It is used to evaluate the signal denoising performance of the proposed filter model. We have also evaluated the proposed filter's performance for two different pathological PCG signals of 2 ms duration taken from the PhysioNet database [55, 56] in the presence of Gaussian noise. The proposed filter output is compared to other recently proposed cascaded filter models objectively in terms of MSE, SNR, ANR, PSNR [57, 58], correlation coefficient (CC) [59, 60], and Mean Absolute Error (MAE) and subjectively in terms of the output signal quality. Simulation parameters are as follows: filter length *M* = 2; the fixed step size used for the adaptive filter is 0.01. The value of parameter *k* is selected as two. The value of *ρ*_threshold_ is appropriately selected depending on the input SNR level, noise added, and output desired. Simulation is conducted in MATLAB version 2017b to extract the clean signal from the noise-corrupted signal.

## 4. Performance of Proposed Variable Stage Cascaded SE LMS Adaptive Filter for the Fetal PCG Signals

### 4.1. Subjective Performance Evaluation

The subjective performance evaluation of the proposed Variable Stage Cascaded SE LMS adaptive filter in output signal quality is depicted below. Two different noises are added to the signal, and the performance of the proposed filter is noted in the presence of Gaussian and pink noise.

- *Gaussian Noise Environment*. The restoration of clean fetal PCG signal deteriorated by Gaussian noise of input SNR = +4 dB is shown in Figure 4. We infer from Figure 4(d) that the replica of the clean signal is obtained at stage 3 using the proposed filter model.  Figure 5 depicts the progressive restoration of the signal at stages 1, 2, and 3. As depicted in Figures 5(b)–5(d), the signal is more corrupted by the noise at stage 1, and progressively, the noise reduces by adding more stages. The best estimate of the clean signal is achieved at stage 3. In Figure 6, the output of the proposed filter is compared with the conventional Sign Error LMS filter and the existing 2-stage [49] and 3-stage [50] cascaded adaptive filter models. We have also illustrated the performance of the proposed filter model by using a fixed step size for all the stages in Figure 6(e).  Figure 7 depicts a high noise scenario where the Gaussian input noise level is set as −4 dB input SNR. As observed in Figure 7(d), the proposed filter performs efficiently and accurately estimates the clean signal even in high noise conditions.  Figure 8 shows progressive restoration of the clean fPCG signal at each consecutive stage. This shows that the performance of the proposed VS Cascaded SE LMS Adaptive Filter is better as we increase the number of stages, and as noted in Figure 8(d) at stage 3, the fetal PCG signal is restored with minimum noise. In Figure 9, the performance of the proposed filter for fPCG signal denoising in high noise conditions is compared with the other filter models.
- *Pink Noise Environment*. The performance of the proposed filter should be validated in the presence of pink noise, which represents the colored noise scenario. The clean signal is corrupted by the pink noise of input SNR = +4 dB, as depicted in Figure 10(c). Restoration of clean signal with minimum noise is attained using the proposed filter model as depicted in Figure 10(d).  Figure 11 shows the performance of the proposed VS Cascaded SE LMS Adaptive Filter at each stage. It can be noted that, at stage 3, the fPCG signal is restored with minimum noise.  Figure 12 shows the comparison of the output of existing filter models with the proposed filter. The performance of the proposed filter in a high noise environment is depicted in Figure 13, where the input pink noise level is −4 dB. From Figure 13(d), it is evident that the proposed filter model is effective in minimizing colored noise.  Figure 14 shows the stagewise performance of the proposed VS CASCADED SE LMS Adaptive Filter, and Figure 14(d) infers that the fPCG signal is restored with minimum noise at stage 3. The performance of the proposed filter is compared with other existing filter models at high input noise levels in Figure 15.

### 4.2. Objective Performance Evaluation

In Table 1, the relationship between MSE and correlation between *e*_*i*_(*n*) and *v*′(*n*) is depicted at each stage. Column 6 of Table 1 shows the different step sizes for each stage. The clean fPCG signal taken from SUFHSDB corrupted by Gaussian and pink noise of input SNR +4 and −4 dB is used to test the performance of the proposed filter. In the field of biomedical engineering, the accuracy of the result is a major criterion for evaluating an algorithm [61, 62] which is verified by objective evaluation. The objective comparison of the proposed filter output with the conventional SE LMS filter and existing 2-stage and 3-stage cascaded filter models is performed in terms of MSE, SNR, ANR, PSNR, CC, and MAE. The results are tabulated in Table 2.

## 5. Performance of Proposed Variable Stage Cascaded SE LMS Adaptive Filter for the Pathological PCG Signals

### 5.1. Subjective Performance Evaluation

The subjective performance evaluation of the proposed Variable Stage Cascaded SE LMS adaptive filter is depicted below. Two pathological PCG signals (a0001 and a0115) taken from the PhysioNet database are corrupted by Gaussian noise, and the denoising performance of the proposed filter is noted. The restoration of clean pathological PCG signal from records a0001 and a0115 deteriorated by Gaussian noise of input SNR = +5 dB is shown in Figures 16 and 17, respectively. It is noted from Figures 16(d) and 17(d) that the best estimate of the clean signal is obtained at stage 3 using the proposed filter model. The denoising performance of the proposed filter model at a high Gaussian input noise level of −5 dB SNR is depicted in Figures 18 and 19. We note from Figures 18(d) and 19(d) that, for both the pathological signals (a0001 and a0115), the proposed filter gives an accurate estimate of the clean signal.

### 5.2. Objective Performance Evaluation

In Table 3, we have compared the performance of the proposed filter model with other cascaded filter models in terms of MSE, SNR, ANR, PSNR, CC, and MAE for both pathological signals (a0001 and a0115) corrupted by Gaussian noise.

### 5.3. Computational Complexity

The number of multiplications and additions required in one iteration of the algorithm decides the computational complexity.  Table 4 presents the number of computations required for the proposed VS Cascaded SE LMS Adaptive Filter model compared to the other recently proposed filter models for Adaptive Noise Cancellation.

## 6. Discussion

### 6.1. Performance of Proposed Variable Stage Cascaded SE LMS Adaptive Filter for the Fetal PCG Signals

#### 6.1.1. Subjective Performance Evaluation

In this work, we have proposed an Adaptive Noise Canceller based on the SE LMS algorithm for PCG signal denoising. We have implemented an automatic adjustment of the number of cascaded stages and step size for each stage. We have compared our results with the 2-stage cascaded ANC structure proposed in [49] and with 3-stage cascaded ANC structure proposed in [50]. Also, we have used a fixed step size for the filter at all stage ANCs and compared the results with the proposed self-adjustable step-size filter model.

- *Gaussian Noise Environment*. Figures 4 and 5 depict the efficient denoising performance of the proposed filter model in the presence of Gaussian noise of input SNR level +4 dB. From Figure 6, we infer that, compared with the current filter outputs, the proposed filter model with variable step size for each stage reduces the noise more efficiently and at high speeds, as proved in Figure 6(f). Figures 7 and 8 depict the remarkable performance of the proposed filter model in the presence of Gaussian noise of input SNR level −4 dB. We note that, compared to Figures 9(b)–9(e), Figure 9(f) provides better signal denoising, which indicates that the proposed filter with variable step size for each stage is more effective in eliminating the noise signals.
- *Pink Noise Environment*. The proposed filter exhibits good denoising properties in nonstationary noise, as noted in Figures 10 and 11 in the presence of pink noise.  Figure 12(f) shows that the proposed filter successfully recovers the clean signal with reduced noise. Even if the noise levels are high, the proposed filter model performs efficiently well, as depicted in Figures 13 and 14. It is noted in Figures 15(b)–15(f) that, compared with the existing filters, the proposed filter exhibits better denoising capability. The variable step size for each stage also reduces the noise levels compared to the fixed step size for all the stages. It concludes that the proposed Variable Stage Cascaded SELMS adaptive filter has the best noise reduction capability and proves to be very attractive in biomedical for denoising PCG signals corrupted by Gaussian and colored noises. We also infer from the subjective analysis that the proposed filter model reduces the Gaussian noise more effectively than the colored Pink noise.

#### 6.1.2. Objective Performance Evaluation

The proposed adaptive filter structure has a Variable Stage Cascaded SE LMS adaptive filter configuration with different step sizes for each stage. The number of stages to be cascaded is controlled automatically depending on the correlation between the output error signal of each stage ANC and the reference input noise signal at stage I ANC. As observed from Table 1, the correlation between *e*_1_(*n*) and *v*′(*n*) is higher than the correlation between *e*_3_(*n*) and *v*′(*n*). This means that as we increase the number of cascaded stages, the estimate of a clean signal at the error output of ANC *e*_*i*_(*n*) is less related to the noise signal and replicates the clean signal, thus reducing the MSE value. Consider the case of speech signal corrupted by Gaussian noise of input SNR = −4 dB. As it can be observed from Table 1, as the correlation *ρ*_*e*_3_(*n*)*v*′_ drops from 0.0144 at stage II to 0.0123 at stage III, the MSE value also reaches a minimum value of 2.03*E* − 05 at stage III. Hence, it is concluded that the MSE value keeps reducing if more number of stages are cascaded since *ρ*_*e*_*i*_(*n*)*v*′_ is lesser as the number of stages *i* is increased. The value of *ρ*_threshold_ is selected depending on the type of noise, input noise level, and output MSE, SNR values desired. The value of *ρ*_threshold_ decides the number of filter stages to be cascaded, and this *ρ*_threshold_ value can be found by the trial and error method. The adaptive filter at each stage ANC requires a different step size. This is because the reference input signal to the adaptive filter at stage I is a noise signal *v*′(*n*) correlated to the additive noise *v*(*n*). And the reference input signal to the consecutive stage adaptive filter is the difference between the input and output signal of the previous stage adaptive filter *x*_*i*_(*n*)=*x*_*i*−1_(*n*) − *y*_*i*−1_(*n*). Thus, the maximum bound on the step size *μ*_max_ changes depending on the input signal. We either multiply or divide the previous stage step-size value by a constant “*k*” to obtain the next stage's step size. In this case, the fixed step size at stage 1 is assumed to be 0.01, and the value of “*k*” is selected as 2. The maximum bound on step size increases at each stage. Therefore, we multiplied the step size of the previous stage by a factor of 2 to obtain the step size of the next stage. This provides optimal performance in terms of MSE, as noted in Table 1. Both *ρ*_threshold_ and “*k*” values are determined using the trial and error method, which is the only drawback in the proposed filter model. Table 2 concludes that the proposed filter gives the minimum MSE values for both the noise signals at different input noise levels. At the same time, we also infer that the proposed Variable Stage Cascaded SELMS adaptive filter model gives better performance in Gaussian noise than pink noise environment. The proposed filter outperforms the existing 2-stage and 3-stage cascaded filter models in terms of MSE, SNR, ANR, PSNR, MAE, and CC. The proposed adaptive filter structure gives an output SNR value of at least 10 dB higher than the existing cascaded adaptive filters in a Gaussian noise environment and 2 dB higher output SNR values in the presence of colored noise. In the presence of Gaussian noise, the Peak SNR values are 7 dB higher, and for pink noise, the improvement is 1-2 dB. The average noise reduction is around 10–12 dB improved for Gaussian noise and 1-2 dB higher for pink noise denoising. The proposed filter model reduces Mean Absolute Error values and improves the correlation coefficient between the clean signal and its estimate.

## 7. Performance of Proposed Variable Stage Cascaded SE LMS Adaptive Filter for the Pathological PCG Signals

### 7.1. Subjective Performance Evaluation

From Figures 16–19, it is evident that the proposed filter model performs well in the presence of different levels of Gaussian noise and gives excellent denoising of both pathological signals.

### 7.2. Objective Performance Evaluation

Table 3 infers that the proposed filter model provides an SNR value of 10–15 dB higher than the existing cascaded adaptive filter models for denoising pathological signals. The average noise reduction capability is also 10 dB higher than the existing filter models. The Peak SNR values are improved by 6 dB, and MSE values reduce by 75–80%. There is a reduction of 70–72% in the Mean Absolute Error, and the correlation between the clean signal and its estimate is also high.

### 7.3. Computational Complexity

We have employed an adaptive filter-based ANC system for fPCG and pathological PCG signal denoising in this work. Adaptive noise cancellers are primarily used to remove noise from speech and audio signals, and we have explored their usage for denoising PCG signals. The main idea is to reduce the computational time and complexity to build cost-effective hardware for recording heart signals without noise. Therefore, we compare the computational complexity of the proposed filter model with other recently proposed filter models for Adaptive Noise Cancellation in various fields. From Table 4, we infer that the conventional SE LMS filter requires a minimum number of computations. The total multiplications and additions for each stage are *M* + 1, where *M* is the filter order. Therefore, we have employed an SE LMS adaptation algorithm for the filters in all cascaded ANC stages. The total number of computations required for the proposed filter model depends on the number of stages used; the cascaded stages are *L* = 3 for denoising PCG signals in the presence of Gaussian and pink noise. The proposed filter model introduces additional computations to automatically select the number of cascaded stages (based on the correlation coefficient) and different step size for each stage (based on the autocorrelation matrix). We have emphasized that a cascaded filter structure is very efficient for an ANC system. Using other filtering techniques apart from SE LMS in a cascaded filter model will lead to a complex structure. Thus, we can conclude that the proposed Variable Stage (VS) Cascaded SELMS Adaptive Filter model provides a cost-effective and straightforward solution for PCG signal denoising in recording heart signals.

## 8. Conclusion

A robust signal denoising scheme is presented in this paper based on a novel multistage cascaded LMS adaptive algorithm. The proposed Variable Stage (VS) Cascaded SELMS Adaptive Filter model in ANC systems offers an improved solution to achieve faster convergence speed and a lower MSE by automatically adjusting the number of filter stages cascaded and the step size for each stage. The simulation performed on fetal PCG and pathological PCG signals concludes that the proposed VS Cascaded SELMS Adaptive Filter outperforms the conventional SELMS and the existing 2-stage and 3-stage cascaded LMS adaptive filter structure, thus improving convergence speed. Also, significantly lower MSE is achieved by the proposed filter model than the conventional SELMS, 2-stage, and 3-stage cascaded LMS filter structures. Cost-effective hardware ANC systems can be implemented using the proposed filter model with simple mathematical modeling.

## Figures and Tables

**Figure 1:** Block representation of ANC.

**Figure 2:** Block diagram of proposed Variable Stage Cascaded SE LMS adaptive filter model.

**Figure 3:** Schematic diagram of proposed Variable Stage Cascaded SE LMS adaptive filter model.

**Figure 4:** Denoising of FPCG signal corrupted by Gaussian noise of input SNR = +4 dB using the proposed VS Cascaded SE LMS Adaptive Filter output. (a) Clean signal. (b) Additive Gaussian Noise signal. (c) Noisy signal. (d) Proposed VS Cascaded SE LMS Adaptive Filter output.

**Figure 5:** Proposed VS Cascaded SELMS Adaptive Filter stagewise restoration of clean signal (Gaussian noise with input SNR = +4 dB). (a) Clean signal. (b) Proposed VS Cascaded SELMS Adaptive Filter stage 1. (c) Output at stage 2. (d) Output at stage 3.

**Figure 6:** Comparison of proposed VS Cascaded SELMS Adaptive Filter output with various filters (fPCG signal with Gaussian noise input SNR = +4 dB). (a) Clean signal. (b) Conventional SE LMS filter output. (c) Existing 2-stage LMS filter output. (d) Existing 3-stage LMS filter output. (e) Proposed VS Cascaded SELMS Adaptive Filter output (fixed step size). (f) Proposed VS Cascaded SELMS Adaptive Filter output (variable step size).

**Figure 7:** Denoising of fPCG signal corrupted by Gaussian noise of input SNR = −4 dB using the proposed VS Cascaded SE LMS Adaptive Filter output. (a) Clean signal. (b) Additive Gaussian Noise signal. (c) Noisy signal. (d) Proposed VS Cascaded SE LMS Adaptive Filter output.

**Figure 8:** Proposed VS Cascaded SELMS Adaptive Filter stagewise restoration of clean signal (Gaussian noise with input SNR = −4 dB). (a) Clean signal. (b) Proposed VS Cascaded SELMS Adaptive Filter stage 1. (c) Output at stage 2. (d) Output at stage 3.

**Figure 9:** Comparison of proposed VS Cascaded SELMS Adaptive Filter output with various filters (fPCG signal with Gaussian noise input SNR = −4 dB). (a) Clean signal. (b) Conventional SE LMS filter output. (c) Existing 2-stage LMS filter output. (d) Existing 3-stage LMS filter output. (e) Proposed VS Cascaded SELMS Adaptive Filter output (fixed step size). (f) Proposed VS Cascaded SELMS Adaptive Filter output (variable step size).

**Figure 10:** Denoising of fPCG signal corrupted by pink noise input SNR = +4 dB using the proposed VS Cascaded SE LMS Adaptive Filter output. (a) Clean signal. (b) Additive Gaussian Noise signal. (c) Noisy signal. (d) Proposed VS Cascaded SE LMS Adaptive Filter output.

**Figure 11:** Proposed VS Cascaded SELMS Adaptive Filter stagewise restoration of clean signal (pink noise with input SNR = +4 dB). (a) Clean signal. (b) Proposed VS Cascaded SELMS Adaptive Filter stage 1. (c) Output at stage 2. (d) Output at stage 3.

**Figure 12:** Comparison of proposed VS Cascaded SELMS Adaptive Filter output with various filters (FPCG signal with pink noise input SNR = +4 dB). (a) Clean signal. (b) Conventional SE LMS filter output. (c) Existing 2-stage LMS filter output. (d) Existing 3-stage LMS filter output. (e) Proposed VS Cascaded SELMS Adaptive Filter output (fixed step size). (f) Proposed VS Cascaded SELMS Adaptive Filter output (variable step size).

**Figure 13:** Denoising of fPCG signal corrupted by pink noise input SNR = −4 dB using the proposed VS Cascaded SE LMS Adaptive Filter output. (a) Clean signal. (b) Additive Gaussian Noise signal. (c) Noisy signal. (d) Proposed VS Cascaded SE LMS Adaptive Filter output.

**Figure 14:** Proposed VS Cascaded SELMS Adaptive Filter stagewise restoration of clean signal (pink noise with input SNR = −4 dB). (a) Clean signal. (b) Proposed VS Cascaded SELMS Adaptive Filter stage 1. (c) Output at stage 2. (d) Output at stage 3.

**Figure 15:** Comparison of proposed VS Cascaded SELMS Adaptive Filter output with various filters (fPCG signal with pink noise input SNR = −4 dB). (a) Clean signal. (b) Conventional SE LMS filter output. (c) Existing 2-stage LMS filter output. (d) Existing 3-stage LMS filter output. (e) Proposed VS Cascaded SELMS Adaptive Filter output (fixed step size). (f) Proposed VS Cascaded SELMS Adaptive Filter output (variable step size).

**Figure 16:** Denoising of pathological PCG signal (a0001) corrupted by Gaussian noise of input SNR = +5 dB using the proposed VS Cascaded SE LMS Adaptive Filter output. (a) Clean signal. (b) Additive Gaussian Noise signal. (c) Noisy signal. (d) Proposed VS Cascaded SE LMS Adaptive Filter output.

**Figure 17:** Denoising of pathological PCG signal (a0001) corrupted by Gaussian noise of input SNR = −5 dB using the proposed VS Cascaded SE LMS Adaptive Filter output. (a) Clean signal. (b) Additive Gaussian Noise signal. (c) Noisy signal. (d) Proposed VS Cascaded SE LMS Adaptive Filter output.

**Figure 18:** Denoising of pathological PCG signal (a0115) corrupted by Gaussian noise of input SNR = +5 dB using the proposed VS Cascaded SE LMS Adaptive Filter output. (a) Clean signal. (b) Additive Gaussian Noise signal. (c) Noisy signal. (d) Proposed VS Cascaded SE LMS Adaptive Filter output.

**Figure 19:** Denoising of pathological PCG signal (a0115) corrupted by Gaussian noise of input SNR = −5 dB using the proposed VS Cascaded SE LMS Adaptive Filter output. (a) Clean signal. (b) Additive Gaussian Noise signal. (c) Noisy signal. (d) Proposed VS Cascaded SE LMS Adaptive Filter output.

**Algorithm 1:** Proposed Variable Stage Cascaded Sign Error LMS adaptive filter.

**Table 1:** Variation of the correlation function and step size at each stage of proposed VS Cascaded SELMS Adaptive Filter for fPCG input signal corrupted by Gaussian and pink noise.

Noise	Input SNR	Stage	MSE	*ρ*_*e*_*i*_(*n*)*v*′(*n*)_	*μ*_*i*_
Gaussian	+4 dB	I	5.70*E* − 05	0.0234	0.01
		II	2.27*E* − 05	0.016	0.02
		III	1.04*E* − 05	0.0116	0.04
	−4 dB	I	8.67*E* − 05	0.0161	0.01
		II	3.88*E* − 05	0.0144	0.02
		III	2.03*E* − 05	0.0123	0.04

Pink	+4 dB	I	1.72*E* − 04	0.014	0.01
		II	1.45*E* − 04	0.0043	0.02
		III	1.36*E* − 04	0.0001	0.04
	−4 dB	I	2.98*E* − 04	0.0192	0.01
		II	2.50*E* − 04	0.0014	0.02
		III	2.36*E* − 04	0.0001	0.04

**Table 2:** Comparison of MSE, SNR, ANR, PSNR, CC, and MAE performance of the proposed VS Cascaded SELMS Adaptive Filter with the various existing filter models for fPCG signals.

Noise	Input SNR	Filter Structure	MSE	SNR (dB)	ANR (dB)	PSNR (dB)	CC	MAE
Gaussian	+4 dB	Conventional SELMS adaptive filter	5.45*E* − 05	45.5658	50.6788	42.2838	0.9946	0.002
		Existing 2-S cascaded LMS adaptive filter	3.58*E* − 05	50.2054	50.3086	44.49	0.9967	0.0017
		Existing 3-S cascaded LMS adaptive filter	2.71*E* − 05	52.9885	53.0913	45.6369	0.9975	0.0015
		Proposed VS Cascaded SELMS Adaptive Filter (FSS)	2.59*E* − 05	53.1973	53.2649	45.7548	0.9976	0.0011
		Proposed VS Cascaded SELMS Adaptive Filter (VSS)	1.04*E* − 05	62.5934	62.6348	49.0503	0.9989	7.42*E* − 04

Gaussian	−4 dB	Conventional SELMS adaptive filter	8.14*E* − 05	41.8965	51.0083	40.7003	0.9923	0.0024
		Existing 2-S cascaded LMS adaptive filter	3.70*E* − 05	49.8859	49.9992	43.8492	0.9962	0.0018
		Existing 3-S cascaded LMS adaptive filter	3.01*E* − 05	51.9602	52.0741	45.4376	0.9974	0.0016
		Proposed VS Cascaded SELMS Adaptive Filter (FSS)	3.91*E* − 05	48.0708	48.1802	43.4126	0.9958	0.0019
		Proposed VS Cascaded SELMS Adaptive Filter (VSS)	2.03*E* − 05	55.8844	55.9548	47.7843	0.9985	9.74*E* − 04

Pink	+4 dB	Conventional SELMS adaptive filter	1.72*E* − 04	34.5489	34.8672	37.6559	0.9845	0.0096
		Existing 2-S cascaded LMS adaptive filter	1.63*E* − 04	35.0507	35.3253	37.8738	0.9852	0.0094
		Existing 3-S cascaded LMS adaptive filter	1.58*E* − 04	35.4005	35.6751	38.0257	0.9857	0.0093
		Proposed VS Cascaded SELMS Adaptive Filter (FSS)	1.47*E* − 04	36.1219	36.3434	38.339	0.9867	0.009
		Proposed VS Cascaded SELMS Adaptive Filter (VSS)	1.36*E* − 04	37.0542	37.0618	38.657	0.9876	0.0087

Pink	−4 dB	Conventional SELMS adaptive filter	2.98*E* − 04	29.0166	29.5294	35.2532	0.9731	0.0124
		Existing 2-S cascaded LMS adaptive filter	2.64*E* − 04	30.2438	30.5464	35.7862	0.9761	0.012
		Existing 3-S cascaded LMS adaptive filter	2.63*E* − 04	30.2934	30.5959	35.8077	0.9762	0.012
		Proposed VS Cascaded SELMS Adaptive Filter (FSS)	2.54*E* − 04	30.6067	30.8777	35.9438	0.9769	0.0117
		Proposed VS Cascaded SELMS Adaptive Filter (VSS)	2.36*E* − 04	31.349	31.5948	36.2661	0.9786	0.0114

**Table 3:** Comparison of MSE, SNR, ANR, PSNR, MAE, and CC performance of the proposed VS Cascaded SELMS Adaptive Filter with the various existing filter models for pathological PCG signals.

Record	Noise	Input SNR	Filter structure	MSE	SNR (dB)	ANR (dB)	PSNR (dB)	MAE	CC
a0001	Gaussian	+5 dB	Conventional SELMS adaptive filter	7.59*E* − 05	21.6266	26.2004	41.1998	0.0052	0.9467
			Existing 2-S cascaded LMS adaptive filter	9.40*E* − 05	19.4818	21.3908	40.2684	0.0069	0.9352
			Existing 3-S cascaded LMS adaptive filter	6.85*E* − 05	22.651	24.5485	41.6447	0.0051	0.9517
			Proposed VS Cascaded SELMS Adaptive Filter (FSS)	3.71*E* − 05	28.7909	29.5316	44.3113	0.0032	0.9731
			Proposed VS Cascaded SELMS Adaptive Filter (VSS)	1.66*E* − 05	36.8464	37.4117	47.8097	0.0017	0.9877

a0001	Gaussian	−5 dB	Conventional SELMS adaptive filter	1.03*E* − 04	18.5649	28.4198	39.8702	0.0044	0.9308
			Existing 2-S cascaded LMS adaptive filter	1.07*E* − 04	18.2324	20.1592	39.7258	0.0056	0.9259
			Existing 3-S cascaded LMS adaptive filter	6.50*E* − 05	23.1706	25.2832	41.8704	0.0032	0.9545
			Proposed VS Cascaded SELMS Adaptive Filter (FSS)	5.34*E* − 05	25.1399	26.2376	42.7257	0.0027	0.9621
			Proposed VS Cascaded SELMS Adaptive Filter (VSS)	2.35*E* − 05	33.3264	33.9951	46.281	0.0015	0.9826

a0115	Gaussian	+5 dB	Conventional SELMS adaptive filter	1.09*E* − 04	27.3987	32.2008	39.6225	0.0046	0.9692
			Existing 2-S cascaded LMS adaptive filter	9.14*E* − 05	29.1654	30.0147	40.3897	0.0052	0.9741
			Existing 3-S cascaded LMS adaptive filter	6.12*E* − 05	33.1816	34.0441	42.1339	0.0031	0.9825
			Proposed VS Cascaded SELMS Adaptive Filter (FSS)	5.36*E* − 05	34.5118	34.928	42.7116	0.0029	0.9845
			Proposed VS Cascaded SELMS Adaptive Filter (VSS)	2.26*E* − 05	43.1482	43.4444	46.4624	0.0016	0.9934

a0115	Gaussian	−5 dB	Conventional SELMS adaptive filter	1.66*E* − 04	23.2246	32.9978	37.8097	0.0043	0.9544
			Existing 2-S cascaded LMS adaptive filter	9.49*E* − 05	28.791	29.6225	40.2271	0.0035	0.973
			Existing 3-S cascaded LMS adaptive filter	6.49*E* − 05	32.5952	33.4509	41.8793	0.0022	0.9814
			Proposed VS Cascaded SELMS Adaptive Filter (FSS)	7.83*E* − 05	30.7113	31.3171	41.0611	0.0027	0.9776
			Proposed VS Cascaded SELMS Adaptive Filter (VSS)	3.12*E* − 05	39.9183	40.3421	45.0596	0.0015	0.9909

**Table 4:** Computational cost of proposed filter model in comparison with the other adaptive filtering algorithms.

Filter structure	‘∗'or‘/'	‘+'or‘−'
LMS adaptive algorithm [63]	2*M* + 2	2*M*
NLMS adaptive algorithm [64]	3*M* + 3	3*M*
FxLMS adaptive algorithm [65]	3*M* + 1	3*M* − 2
Affine Projection Algorithm [66]	2*P*^2^ + 2PM + *M*	2*P*^2^*M* + PM-*P*^2^
RLS Algorithm [67]	3*M*^2^+4*M*+1	3*M*^2^+4*M*
Proposed VS Cascaded SE LMS Adaptive Filter	*L*(*M* + 1)	*L*(*M* + 1)

## Data Availability

Data were taken from the PhysioNet database. (https://doi.org/10.13026/42eg-8e59).
